RETRACTED

# Application Analysis of UPOINT System in Chinese Type III Prostatitis Patients: A Single Center Experience

**DOI:** 10.1155/2022/9227032

**Published:** 2022-05-02

**Authors:** Zhongxiao Zhang, Xiaonan Su, Chengfeng Cai, Zehua Wang

**Affiliations:** ^1^Department of Urology, Qilu Hospital (Qing Dao), Shandong University, Qingdao, Shandong 266000, China; ^2^Department of Urology, Zoucheng People's Hospital, Zoucheng, Shandong 273500, China; ^3^Department of Urology, Qilu Hospital, Cheeloo College of Medicine, Shandong University, Jinan, Shandong 250014, China; ^4^Department of Urology, Qilu Hospital, Shandong University, Jinan, Shandong 250012, China

## Abstract

**Objective:**

UPOINT clinical phenotype system was used to estimate the type III prostatitis patients. Put in the erectile dysfunction (ED) domain and analysis the ED domain's effect towards the UPOINT system.

**Methods:**

A total of 126 patients with type III prostatitis were prospectively collected and classified in each domain of the UPOINT system, including urinary, psychosocial, organ-specific, infection, neurological/systemic, and tenderness. Symptom severity was measured using the national institutes of health chronic prostatitis symptom index (NIH-CPSI) and the international prostate symptom score (IPSS). The erectile function was evaluated using the international index of erectile function (IIEF-5). Mental state was evaluated using the Symptom Checklist 90 (SCL-90). The quality of life of patients was assessed by the Quality of Life scale (QoL).

**Results:**

The percentage of patients positive for each domain was 60.32%, 43.65%, 53.17%, 11.11%, 42.06%, and 33.33% for the urinary, psychosocial, organ-specific, infection, neurological/systemic, and tenderness, respectively. There were significant correlations between the number of positive UPOINT domains and total NIH-CPSI (*r* = 0.630, *P* < 0.001) and IPSS (*r* = 0.429, *P* < 0.001). Symptom duration was associated with a number of positive domains (*r* = 0.194, *P* < 0.05). After adding an ED domain to establish a modified UPOINT system, the correlation between the number of positive domains and symptom severity was not improved (0.630 to 0.590, *P* < 0.001). The percentage of the patients who suffered psychosocial problems was 43.65%.

**Conclusions:**

In our cohort, the number of positive domains was correlated with symptom severity. Inclusion of the ED phenotype in the UPOINT phenotype classification system did not significantly enhance the association of positive presentation with symptom severity. Our findings presented do not support the utility of using ED as a stand-alone item in the UPOINT domain. Psychological problems should be considered when treating type III prostatitis patients.

RETRACTED

## 1. Introduction

Prostatitis is one of the common diseases of adult men. According to the new classification method of National Institutes of Health (NIH) in 1995 [1, 2], type III prostatitis is chronic prostatitis/chronic pelvic pain syndromes (CP/CPPS), which is also a very common type of prostatitis and can reach 90% of the patients concerned. Long-term and repeated pelvic pain and discomfort, lasting more than 3 months, may be accompanied by different degrees of lower urinary tract symptoms (LUTS) and erectile dysfunction (ED), which are the main symptoms of patients with type III prostatitis. About 15.0%-48.3% of patients with type III prostatitis have erectile dysfunction (ED) [3, 4], and ED will significantly affect the symptoms and quality of life of patients. In 2009, Shoskes et al. [5] established a six item system based on clinical phenotype-UPOINT to classify patients with type III prostatitis and interstitial cystitis and guide the selection of treatment options. However, Shockers did not add ED as an independent phenotype to the UPOINT system. Whether ED should be incorporated into UPOINT system has been controversial [6, 7]. The initial description of psychosocial in the UPOINT system is also vague. At present, there is no exact score to regulate whether the P phenotype is positive or not. Therefore, we used the UPOINT phenotypic classification system to classify and evaluate some Chinese patients with type III prostatitis and continue to study the impact of psychosocial symptoms and ED on UPOINT system.

## 2. Material and Methods

### 2.1. Clinical Data

A total of 126 patients diagnosed with type III prostatitis by the same doctor from July 2015 to November 2019 were collected. All patients enrolled in this study were informed and signed the informed consent.

### 2.2. Inclusion Criteria and Exclusion Criteria

Inclusion criteria were as follows: ① the diagnosis of type III prostatitis was carried out according to the 2014 Chinese Guidelines for the Diagnosis and Treatment of Urological Diseases, combined with the NIH diagnostic criteria; ② all patients signed the informed consent. Exclusion criteria were as follows: ① patients without normal sexual life; ② patients with congenital organ dysplasia.

### 2.3. Research Methods

1. Basic patient information is collected, including general characteristics of patients, age, height, weight, etc.
2. The patient was examined for the following items, including prostate surgery examination and expressed prostatic secretious (EPS). Urinary bacterial culture was performed by using a two-cup method
3. The following questionnaires were used: National Institutes of Health Chronic Prostatitis Symptom Index (NIH-CPSI); International Prostate Symptom Score (IPSS); International Index of Erectile Function (IIEF-5); Symptom Checklist 90 (SCL-90); and Quality of Life (QoL). Symptom severity was measured using the NIH-CPSI and IPSS. The erectile function was evaluated using the IIEF-5. Mental state was evaluated using the SCL-90. The quality of life of patients was assessed by the Quality of Life scale (QoL)
4. UPOINT phenotypes were diagnosed. UPOINT has 6 phenotypes. The six phenotypes were urinary, psychosocial, organ specific, infection, neurological/systemic, and tenderness of pelvic floor muscle. The number of positive phenotypes was significantly correlated with the symptom index of chronic prostatitis (NIH-CPSI)

RETRACTED

### 2.4. Ethical Review and Informed Consent

The study was approved by the Qilu Hospital committee on human research. Before the answer sheet, explain the purpose of this study to the patients under investigation and clarify that the results will be treated confidentially, and personal privacy will not be revealed, so as to obtain patients' understanding and consent.

### 2.5. Statistical Treatment

All data were collected using SPSS 23.0 statistics software processing data. The mean ± standard deviation and median were used to statistically express the basic data. Spearman correlation analysis was used to study the correlation between UPOINT and other measurement data such as NIH-CPSI score and IPSS score; rank sum test was used to compare the differences of symptom score and quality of life among different factor numbers, and rank sum test was used to test the differences of symptom severity and quality of life among positive and negative factors of UPOINT; the correlation coefficient after adding ed phenotype was compared with that without adding ed phenotype by *Z*-test.

## 3. Result

### 3.1. Baseline Data

In this questionnaire survey, 130 questionnaires were distributed, and 126 valid questionnaires were recovered, with an effective recovery rate of 96.92%. The basic data scores of 126 patients with type III prostatitis involved in the effective recovery questionnaire are shown in Table 1. There were 34 patients with type IIIA prostatitis and 92 patients with type IIIB prostatitis. The pH value of EPS in patients with type IIIA was 7.17 ± 0.22, with a median of 7.10; the pH value of type IIIB patients was 6.62 ± 0.31, and the median was 6.60. There was significant difference between the two (*t* = 9.412, *P* < 0.001). There was no significant difference in NIH-CPSI score between IIIA patients and IIIB patients (*t* = 0.465, *P* = 0.643).

The proportion of subitem positive factors (1-6) of the UPOINT phenotypic system is as follows: only 1 item is positive (28 cases, 22.22%), 2 items (53 cases, 42.06%), 3 items (19 cases, 15.08%), 4 items (16 cases, 12.70%), 5 items (8 cases, 6.35%), and 6 items (2 cases, 1.59%).

RETRACTED

There was no significant correlation between the number of UPOINT positive factors and the age of patients (*r* = 0.044, *P* = 0.622); there was a positive correlation with the duration of the disease (*r* = 0.194, *P* = 0.029) and no significant correlation with the height of the patient (*r* = −0.009, *P* = 0.919); there was no significant correlation with body weight (*r* = 0.056, *P* = 0.535); there were 31 patients whose BMI index exceeded 25. There was no significant difference between BMI index greater than 25 and NIH-CPSI score (*t* = 0.606, *P* > 0.10).

### 3.2. Analysis of the Relationship between UPOINT and NIH-CPSI

The number of positive factors in UPOINT system showed obvious correlation with NIH-CPSI score (*r* = 0.630, *P* < 0.001), as shown in Figure 1. The relationship between the positivity of each factor and the total score of NIH-CPSI and each subitem score is shown in Table 2. Analysis of the relationship between NIH-CPSI total score and subitems and the number of positive factors of UPOINT shows that the total score and subitems of NIH-CPSI in patients with positive factors are basically higher than those in patients with negative factors.

### 3.3. Analysis of the Relationship between UPOINT and IPSS

IPSS symptom score: most patients showed mild to moderate symptoms, as shown in Table 3. With the increase of the number of UPOINT positive factors, the IPSS score also increased (5 phenotypic positives combined with 6 phenotypic positives), as shown in Figure 2. The Spearman correlation coefficient between the number of UPOINT positive phenotypes and IPSS score was 0.429, *P* < 0.01.

### 3.4. Analysis of the SCL-90 Scale

The scores of each subitem of the total SCL-90 score in patients with type III prostatitis were compared with the national adult norm, showing significant differences. It is suggested that the mental and psychological conditions of patients with type III prostatitis are not good, as shown in Table 4. The SCL-90 score was positively correlated with the number of UPOINT positive factors (*r* = 0.528, *P* < 0.01), and the SCL-90 score was positively correlated with the NIH-CPSI score (*r* = 0.239, *P* < 0.01).

### 3.5. Analysis of the Effect on UPOINT after the Addition of the ED Score

The sample size was 110 cases after excluding those that did not meet IIEF-5 inclusion criteria. There were 55 patients with ED positive (50.00%). There was no significant difference in NIH-CPSI scores between the patients with ED positive and those with ED negative, but there was a difference in SCL-90 scores (*t* = 2.52, *P* < 0.05), and there was no significant difference in QoL scores, as shown in Table 5. There were significant differences in the number of positive phenotypes of UPOINT (*t* = 2.91, *P* = 0.004).

RETRACTED

After ED is included as an independent factor in UPOINT system, the number of UPOINT positive factors is still correlated with NIH-CPSI score (*r* = 0.590, *P* < 0.001). As shown in Figure 3, 6 positive factors and 7 positive factors have been combined. However, when the ED phenotype was not added (*r* = 0.656 > 0.590, *P* < 0.001). The difference between the two coefficients is (*Z* = −2.31, *P* = 0.02); so, the correlation has not been improved after adding ED as an independent phenotype to UPOINT.

## 4. Discussion

### 4.1. General Patient Characteristics

The average age of 126 patients was 32.08 ± 9.57 years old. Most of the patients were in the middle-aged and young age group. This is also in line with the characteristics that type III prostatitis is a common and frequently occurring disease in young adults. A domestic study also shows that most patients with type III prostatitis are younger than 40 years old [6]. Compared with some foreign studies [1], this age composition is still small. The age difference compared with foreign studies may be caused by patients' attention to diseases, daily living habits, economic status, etc. Specific and clear reasons still need large-scale research and investigation to draw conclusions. The average height of 126 patients was 173.75 ± 5.47 cm, the average weight was 69.87 ± 11.17 kg, and the BMI index was 23.14 ± 3.45. According to the WHO classification standard, BMI index greater than 25 is overweight. In this study, 31 of 126 patients were overweight or obese. Whether BMI index exceeds 25 has no significant correlation with NIH-CPSI score (*t* = 0.606, *P* > 0.10). Thus, overweight or obesity may not be one of the influencing factors of type III prostatitis. There was significant difference in the pH value of EPS between patients with type IIIA and patients with type IIIB (*t* = 9.412, *P* < 0.001). The pH value of patients with type IIIA was significantly higher than that of patients with type IIIB. This is consistent with the research results of Meihua et al. [8]. The difference in pH content is mainly caused by the change of citric acid concentration in EPS [9]. In type IIIA patients, the increase of pH value may be due to tissue edema caused by prostatic inflammation, resulting in microcirculation disorder and hypoxia in the tissue. Therefore, the prostate has an obstacle to secretory function, which further reduces the production of citric acid and increases the pH value.

RETRACTED

### 4.2. Analysis of the UPOINT System

Among 126 patients, most patients have two or more phenotypes positive, and different patients often show different clinical symptoms; so, it is not advisable to adopt the same treatment measures, which may also lead to poor long-term curative effect of patients. The number of positive factors in U-UPOINT system has a significant positive correlation with NIH-CPSI score and IPSS score (*r* = 0.630, *P* < 0.01) (*r* = 0.429, *P* < 0.01). The number of phenotypic positive factors can well reflect the severity of symptoms, evaluate patients' symptoms, and effectively formulate individualized treatment plan for patients [10]. Similar to the results of previous studies [4], we also found that the number of positive phenotypes of UPOINT system increased with the increase of symptom duration, regardless of age. These results also indirectly prove that pelvic floor muscle spasm and peripheral nerve changes caused by the initial inflammation of prostate may last for a long time, even after the initial inflammation symptoms are eliminated [11]. In the comparison between NIH-CPSI subscore and UPOINT six phenotypes, we can see that the positivity of the six phenotypes is correlated with NIH-CPSI score, indicating that the six phenotypes are closely related to the severity of symptoms of type III prostate.

### 4.3. Analysis of whether the Erectile Dysfunction Phenotype Can Be Added to the UPOINT

There are many patients with type III prostatitis who suffer from ED symptoms at the same time, and patients with type III prostatitis are also more likely to suffer from ed. A recent foreign large sample survey [12] showed that the number of patients with type III prostatitis in 3194 patients with ED was significantly higher than that in the control population (8.6% vs. 2.5%, *P* < 0.001). Further multiple regression analysis showed that type III prostatitis was an independent risk factor for ED, and the odds ratio of ED in patients with type III prostatitis was 3.62. It is suggested that the risk of ED in patients with type III prostatitis is 3.62 times higher than that in patients without prostatitis. Based on the results of a large sample study, Magri et al. [7] inferred that after ED was added to UPOINT phenotype system, individualized comprehensive treatment may obtain better curative effect. A recent prospective study based on Chinese patients also showed support for adding ed to UPOINT system to improve the efficiency of UPOINT diagnosis and treatment [13]. However, according to the research results of Samplaski [6] and Hedelin [14], the inclusion of ED phenotype cannot enhance the relationship between UPOINT system and NIH-CPSI score and cannot enhance its correlation. Therefore, the inclusion of ED phenotype into UPOINT phenotype system is not supported in our study, we can see that the correlation coefficient did not increase after adding ED phenotype (from 0.656 to 0.590, *P* < 0.001), and whether ED was positive or not had no exact relationship with NIH-CPSI score, no obvious correlation with QoL score, but had correlation with SCL-90 score (*P* < 0.05). The pathogenesis and mechanism of type III prostatitis and ED are unclear, and the symptoms and manifestations are partly coincident, which makes it difficult to distinguish them. Psychological effects, neuroendocrine, arterial system diseases, etc. may all lead to ED, and some of these incentives may also lead to prostatitis, and the symptoms of prostatitis may also aggravate the symptoms of ED. The interaction between the two may form a vicious circle. In this study, whether ED is significantly related to mental and psychological status, and in the statistical process, patients were asked to reflect that the majority of ED cases are secondary to prostatitis. Mental factors become an important bridge between ED and the pathogenic factors of type III prostatitis. The application of SCL-90 may be the reason why the relationship between UPOINT system and NIH-CPSI score cannot be significantly enhanced after ED is added. Different from Magri's research results may be due to different inclusion criteria, mixed outpatient patients with stubborn symptoms, and poor understanding of IIEF-5 score due to patients' low educational level. Whether or not ED can be included in UPOINT has always been controversial. Combined with the results of this study, we temporarily disapprove of including ED in UPOINT system, and whether or not ED can better guide the design of clinical treatment strategies needs further research.

RETRACTED

### 4.4. Analysis of Psychological Factors

In our study, SCL-90 was used to diagnose whether the P phenotype was positive or not, instead of using clinical symptoms to determine whether the P phenotype was positive or not. This greatly reduces the inaccuracy of diagnosis quantification caused by subjective factors of doctors. In the results, we can see that there are 55 patients with SCL-90 with a total score of over 160 or a single score of over 2 or a positive number of over 43 items, accounting for 43.65% of the total cases, far higher than Shoskes' research results [4] It can be seen that the proportion of mental factors in patients with type III prostatitis is quite large. Compared with the national norm [15], we can find that patients with type III prostatitis have obvious mental and psychological problems, among which somatization, compulsion, depression, anxiety, hostility, and psychosis are significantly higher than the norm. These symptoms are also far beyond the psychological symptoms expressed by Shoskes [4]. It can be seen that mental and psychological problems occupy a very important part in patients. There are so many psychological problems in patients with type III prostatitis, which may be caused by the long course of disease, the strong subjective feelings of patients, the poor effect after treatment, and the persistent recovery [16, 17]. This abnormal psychology such as depression, anxiety, hostility, and compulsion will eventually make patients lose confidence in treatment. The symptoms of type III prostatitis are mainly located in the lower abdomen, perineum, and other parts [18]. It is very easy for patients to associate symptoms with sexual function, which further increases the psychological burden of patients and induces psychological problems [19, 20]. Abnormal psychological problems are caused by the symptoms of prostatitis, and mental and psychological problems can adversely affect the patient's body, which not only aggravates the symptoms but also may lead to new symptoms [21]. These situations make us helpless for some patients in clinical diagnosis and treatment. Such common mental and psychological problems in patients with type III prostatitis also suggest that we should comprehensively evaluate the mental and psychological status of patients in clinical diagnosis and treatment. We understand the patient's condition description and psychological characteristics and establish a good doctor-patient trust relationship with the patient, so as to formulate the corresponding treatment plan for the patient.

## 5. Conclusion

In patients with type III prostatitis, the number of positive phenotypes in the UPOINT phenotype classification system was significantly and positively associated with the severity of the symptoms. The inclusion of the ED phenotype did not significantly enhance the association of positive table lines and symptom severity in the UPOINT phenotype classification system, and the results of this study do not support the inclusion of ED in the UPOINT system as an independent phenotype. This study should pay more attention to the mental and psychological problems of patients with type III prostatitis. The patients were all from one hospital; so, the sample size was limited. The lack of a control group in this study is a disadvantage of the study design. There may be errors in the diagnosis of systemic diseases in the UPOINT questionnaire.

RETRACTED

## Figures and Tables

**Figure 1:** CPSI total score of patients with each phenotype of UPOINT. 1 for 1 positive domain, 2 for 2 positive domains, and so on.

**Figure 2:** IPSS score of patients with each phenotype of UPOINT. 1 for 1 positive domain, 2 for 2 positive domains, and so on.

**Figure 3:** CPSI total score of patients with each phenotype of UPOINT. 1 for 1 positive domain, 2 for 2 positive domains, and so on.

**Table 1:** General data of the study subjects.

General information	
Age (years)	32.08 ± 9.57; median 31.00
Height (cm)	173.75 ± 5.47; median 174.00
Weight (kg)	69.87 ± 11.17; median 70.00
BMI index number	23.14 ± 3.45; median 23.46
Duration of the disease course (month)	26.47 ± 35.95; median 12.00
NIH-CPSI (0-43 score)	21.00 ± 6.88
Pain and discomfort (0-21 score)	7.64 ± 4.26
Urination symptoms (0-10 score)	4.40 ± 3.14
Quality of life (0-12 score)	8.96 ± 2.24
IPSS score (points 0-35 score)	10.80 ± 7.73
UPOINT the number of positive cases for each phenotype (*n* (%))	
Urinary (urination)	76 (60.32)
Psychosocial (social mentality)	55 (43.65)
Organ-specific (organ specificity)	67 (53.17)
Infection (infect)	14 (11.11)
Neurologic (neural/system)	53 (42.06)
Tenderness (pelvic floor myalgia)	42 (33.33)
ED(erectile dysfunction)	63 (50.00)

**Table 2:** Relationship between the positive score for each phenotype and the NIH-CPSI total score and the subitem score, ^∗^*P* < 0.05.

UPOINT phenotype	CPSI total scores	Pain and discomfort	Urinary symptoms	Quality of life
Urinary -	17.52 ± 5.29	7.42 ± 3.72	1.60 ± 1.32	8.50 ± 2.35
Urinary +	23.29 ± 6.87	7.79 ± 4.59	6.24 ± 2.59	9.26 ± 2.13
*P* value	*P* < 0.001^∗^	*P* = 0.635	*P* < 0.001^∗^	*P* = 0.067
Psychosocial -	19.73 ± 6.25	7.31 ± 4.03	3.80 ± 2.96	8.62 ± 2.28
Psychosocial +	22.64 ± 7.36	8.07 ± 4.54	5.16 ± 3.24	9.40 ± 2.13
*P* value	*P* = 0.018^∗^	*P* = 0.320	*P* = 0.015^∗^	*P* = 0.049^∗^
Organ-specific -	18.24 ± 5.75	6.00 ± 3.84	3.78 ± 2.83	8.46 ± 2.45
Organ-specific +	23.43 ± 6.91	9.09 ± 4.10	4.94 ± 3.32	9.40 ± 1.95
*P* value	*P* < 0.001^∗^	*P* < 0.001^∗^	*P* = 0.038^∗^	*P* = 0.019^∗^
Infection -	20.75 ± 6.77	7.57 ± 4.28	4.27 ± 3.16	8.91 ± 2.28
Infection +	23.00 ± 7.68	8.21 ± 4.14	5.43 ± 2.95	9.35 ± 1.91
*P* value	*P* = 0.250	*P* = 0.592	*P* = 0.194	*P* = 0.430
Neurologic -	18.95 ± 5.53	6.38 ± 3.70	3.96 ± 2.89	8.60 ± 2.12
Neurologic +	23.83 ± 7.57	9.38 ± 4.39	5.00 ± 3.40	9.45 ± 2.33
*P* value	*P* < 0.001^∗^	*P* < 0.001^∗^	*P* = 0.066	*P* = 0.035^∗^
Tenderness -	19.19 ± 5.66	6.40 ± 3.69	4.19 ± 3.08	8.60 ± 2.20
Tenderness +	24.62 ± 7.71	10.12 ± 4.28	4.81 ± 3.28	9.69 ± 2.17
*P* value	*P* < 0.001^∗^	*P* < 0.001^∗^	*P* = 0.299	*P* = 0.009^∗^

**Table 3:** The International IPSS score of the scale of prostate symptoms.

IPSS grade	Number of people	Percentage (%)
Mild	45	35.71
Moderate	60	47.62
Severe	19	15.08

RETRACTED

**Table 4:** Analysis of the effect on UPOINT after the addition of the ED score, ^∗^*P* < 0.05.

UPOINT result after the addition of the ED score	NIH-CPSI score	QoL score	SCL-90 score
Positive (+)	21.75 ± 7.69	9.00 ± 2.26	137.11 ± 53.09
Negative (-)	20.71 ± 5.83	9.08 ± 2.16	112.27 ± 49.00
*P* value	0.42	0.845	0.013

**Table 5:** Item scores on the SCL-90 scale for patients and the national adult norm, ^∗^*P* < 0.05.

Project	Patient group	Control group	*t*	*P*
Somatization	1.56 ± 0.47	1.37 ± 0.48	4.01	<0.001^∗^
Enforce	1.92 ± 0.69	1.62 ± 0.58	4.33	<0.001^∗^
Interpersonal relation	1.63 ± 0.60	1.65 ± 0.51	-0.298	0.766
Depressed	1.62 ± 0.55	1.50 ± 0.59	2.2	0.030^∗^
Anxious	1.55 ± 0.54	1.39 ± 0.43	2.91	0.004^∗^
Hostilities	1.67 ± 0.66	1.48 ± 0.56	2.93	0.004^∗^
Terrifying	1.27 ± 0.41	1.23 ± 0.41	0.97	0.333
Bigoted	1.44 ± 0.48	1.43 ± 0.57	0.1	0.918
Psychiatric sex	1.47 ± 0.53	1.29 ± 0.42	3.36	0.001^∗^
Total score	142.95 ± 43.85	129.96 ± 38.76	3.04	0.003^∗^

Note: Control group data comes from the national adult norm.

## Data Availability

The labeled dataset used to support the findings of this study are available from the corresponding author upon request.

## References

[1] Xu Y., Zhang L., Shen Y., Yao H., Yong S., You Y. (2020). Effectiveness of psychological interventions for treating chronic prostatitis/chronic pelvic pain syndrome. *Medicine*.

[2] Aktar N., Moudud A., Chen T. (2021). Recent advances in pharmacological interventions of chronic prostatitis/ chronic pelvic pain syndrome. *Current Pharmaceutical Design*.

[3] Liang C. Z., Zhang X. J., Hao Z. Y., Shi H. Q., Wang K. X. (2004). Prevalence of sexual dysfunction in Chinese men with chronic prostatitis. *BJU International*.

[4] Liu L. F., Yang J. R., Yin C., Wang L., He Q. (2008). Current status of cognitive and behavioral patterns of chronic prostatitis among clinicians. *The Chinese Journal of Urology*.

[5] Shoskes D. A., Nickel J. C., Dolinga R., Prots D. (2009). Clinical phenotyping of patients with chronic prostatitis/chronic pelvic pain syndrome and correlation with symptom severity. *Urology*.

[6] Franco J. V., Turk T., Jung J. H. (2019). Non-pharmacological interventions for treating chronic prostatitis/chronic pelvic pain syndrome: a Cochrane systematic review. *BJU International*.

[7] Franco J. V. A., Turk T., Jung J. H. (2019). Pharmacological interventions for treating chronic prostatitis/chronic pelvic pain syndrome. *The Cochrane Database of Systematic Reviews*.

[8] Hui W., Meihua, Xiaozhong Z. (2002). Significance of prostate fluid pH in the diagnosis of chronic prostatitis. *The Journal of Clinical Urology*.

RETRACTED

[9] Brooks D. E., Tate M. E., Mann T., Martin A. W. (1981). Phosphoglycopeptide, a major constituent of the spermatophoric plasma of the octopus (octopus dofleini martini). *Journal of Reproduction and Fertility*.

[10] Paterson C., Kennedy C. (2020). Pharmacological interventions for treating chronic prostatitis/chronic pelvic pain syndrome. *Research in Nursing & Health*.

[11] Breser M. L., Salazar F. C., Rivero V. E., Motrich R. D. (2017). Immunological mechanisms underlying chronic pelvic pain and prostate inflammation in chronic pelvic pain syndrome. *Frontiers in Immunology*.

[12] Chung S. D., Keller J. J., Lin H. C. (2012). A case-control study on the association between chronic prostatitis/chronic pelvic pain syndrome and erectile dysfunction. *BJU International*.

[13] Zhao Z., Zhang J., He J., Zeng G. (2013). Clinical utility of the UPOINT phenotype system in Chinese males with chronic prostatitis/chronic pelvic pain syndrome (CP/CPPS): a prospective study. *PLoS One*.

[14] Hedelin H. H. (2009). Evaluation of a modification of the UPOINT clinical phenotype system for the chronic pelvic pain syndrome. *Scandinavian Journal of Urology and Nephrology*.

[15] Jin H., Wu W., Zhang M. (1986). Preliminary analysis of the SCL-90 assessment results in Chinese normal people. *The Chinese Journal of Neuropsychiatric Disorders*.

[16] Yan Y. (2018). *Effect of Psychological Nursing Intervention and the Quality of Life in Patients with Chronic Prostatitis*.

[17] Xiao H. X., Li L. H., Yang X. Y., Sun Y. T. (2018). *Psychological intervention on improving symptoms and quality of life in patients with chronic prostatitis*.

[18] Wang J., Liang K., Sun H., Li L., Wang H., Cao J. (2018). Psychotherapy combined with drug therapy in patients with category III chronic prostatitis/chronic pelvic pain syndrome: a randomized controlled trial. *International Journal of Urology*.

[19] Gott M. L., Osterdahl P. R., Connors C., Slotman G. (2019). Bariatric surgery does not resolve underlying psychological/behavioral problems in patients with morbid obesity: analysis of 166,601 patients. *Journal of the American College of Surgeons*.

[20] Kim M. J., Kim J., Kho H. S. (2018). Comparison between burning mouth syndrome patients with and without psychological problems. *International Journal of Oral and Maxillofacial Surgery*.

[21] Wazir J., Ullah R., Li S. (2019). Efficacy of acupuncture in the treatment of chronic prostatitis-chronic pelvic pain syndrome: a review of the literature. *International Urology and Nephrology*.

